RETRACTED

# Acupuncture Effect Assessment in APP/PS1 Transgenic Mice: On Regulating Learning-Memory Abilities, Gut Microbiota, and Microbial Metabolites

**DOI:** 10.1155/2022/1527159

**Published:** 2022-04-08

**Authors:** Bo Yang, Min He, Xinhua Chen, Mengmeng Sun, Ting Pan, Xiaohong Xu, Xuesong Zhang, Qing Gong, Ye Zhao, Ziqi Jin, Zedong Cheng

**Affiliations:** ^1^Liaoning University of Traditional Chinese Medicine, No. 79, Chongshan Eastern Rd, Huanggu District, 110847 Shenyang, China; ^2^Changchun University of Chinese Medicine, No. 1035, Boshuo Rd, Jingyue Economic Development District, 130117 Changchun, China; ^3^Northwest University, No. 229, Taibai North Road, Xi' an 710069, China

## Abstract

Alzheimer's disease (AD) is a brain illness that affects learning and memory capacities over time. In recent investigations, acupuncture has been shown to be an effective alternative treatment for AD. We investigated the effect of acupuncture on learning and memory abilities using a water maze in APP/PS1 transgenic mice. The amounts of A*β* and tau protein in mice's hippocampal tissue were determined using Western blot. The levels of IL-1*β*, IL-10, LPS and TNF-*α* in mice's serum were measured using ELISA. The variations of gut microbiota in mice's feces were determined using the 16SrDNA technique, and the metabolites were examined using a untargeted metabolomics methodology. The results showed that acupuncture treatment improved mice's learning and memory abilities substantially. Acupuncture therapy regulated the A*β* and tau protein concentration as well as the levels of IL-10 and LPS. Acupuncture treatment influenced the mouse microbiota and metabolites and had been linked to six biochemical pathways. This study adds to our understanding of the effect of acupuncture on AD and opens the door to further research into the alterations of intestinal bacteria in the presence of AD.

## 1. Introduction

Alzheimer's disease (AD) is a slow-moving neurodegenerative disorder characterized by memory decline, cognitive impairment, and changes in personality. The major neuropathological conditions for the diagnosis of AD are the accumulation of extracellular amyloid *β*-protein (A*β*) as neuroinflammatory plaques and the accumulation of high phosphorylate tau intracellular protein as neurofibrillary tangles [1]. AD is the fourth leading cause of death for people over 65 years of age globally and has become a national public health concern [2]. There is no appropriate cure for AD [3–5], which can only marginally alleviate symptoms such as cognitive control and everyday physical dysfunction, cannot alter the underlying neuropathology or its development, and has some side effects [6–9]. AD patients can lose their capacity to live independently, placing immense pressures on family members, caregivers, and community as a whole. Annual health care costs associated with AD are estimated to be close to 500 billion US dollars [10]. A number of new biological technologies (e.g., genomics, proteomics, and metabolomics) have started to be used in AD research field [11–13]. More and more experiments have demonstrated in recent years that gut microbiota plays an important role in the management of human health and disease through sustaining intestinal homeostasis. [14, 15]. Gut microbiota disorder is linked with multiple disorders, including gastrointestinal diseases [16–19] and AD [20–22]. Gut microbiota has a direct impact on AD, for example, helicobacter pylori enhances tau protein hyperphosphorylation [23]; intestinal disorders can encourage amyloid aggregation, neuroinflammation, oxidative stress, and insulin tolerance in AD pathogenesis [22]; and changes in the composition of gut microbiota can increase the release of lipopolysaccharides (LPSs) and amyloid, which may promote AD pathogenesis [24]. In addition, more and more comparative studies have shown that there are variations in gut microbiota composition between AD patients and healthy people, AD also leads to changes in gut microbiota or is associated with changes in gut microbiota [25–27]. As science offers data and broadens our understanding of AD pathogenesis, the study of gut microbiota provides further opportunities for diagnosis and treatment of AD.

RETRACTED

In the meantime, due to the wide distribution of AD cases globally, more and more complementary and alternative treatments are being used for the care and control of AD [28, 29]. Acupuncture is a common treatment that has been used in the whole world. It is based on the theory and concepts of Chinese medicine and it is healthy, economical, and comfortable and has few side effects [30]. Currently, acupuncture therapy has been commonly used in the care of different diseases, such as pain [31], stroke [32], asthma [33], and gastroenteritis [34]. The use of acupuncture to relieve different symptoms has drawn the interest of scientists all over the world. According to current research findings, the overall regulatory effect of acupuncture on AD can be accomplished by controlling irregular expression of proteins in the brain, by regulating the physiological and pathological status of microglia, mitochondrial autophagy, epigenetic alteration, oxidative activity, and energy metabolism and by enhancing synaptic plasticity [35]. In comparison, acupuncture is usually integrated which is multitargeted and is a systematic and holistic therapy approach that is close to the omics methodology. Omics methods, including proteomics and metabolomics, have been successfully used to screen for disease biomarkers, which is an important technology that makes the acupuncture revolution an important driving force in practice. At present, the study between acupuncture and AD focuses on the rules of acupoint selection and the therapeutic process, and identification indices primarily concentrate on A*β* and tau protein, associated inflammatory factors, dietary factors, neurotransmitters, etc. However, it is important to further investigate whether acupuncture can cure AD, and the biomedical evidence for the treatment of AD. There have been recent research relating the effects of acupuncture to improvements in gut microbiota, investigating the regulatory effects of acupuncture, moxibustion, and electroacupuncture on obesity and ulcerative colitis [36–38], which suggest that gut microbiota could be a potential goal for the therapeutic impact of acupuncture. Therefore, researching the effects of acupuncture combined with controlling the gut microbiota and in vivo treatment of AD may provide a new perspective for understanding acupuncture treatment of AD.

RETRACTED

In this research, acupuncture was used to treat APP/PS1 transgenic mice, which were used as an AD model. Water maze experiments revealed that acupuncture therapy improved the learning and memory capability of the APP/PS1 mice. Acupuncture therapy also had an important effect on the abundance changes of gut microbiota and metabolites of the APP/PS1 mice. Our results suggest that acupuncture, as a holistic approach, has great promise in the treatment and management of AD. This study encourages further research into the effects of acupuncture on variations in the intestinal microbiome associated with AD.

## 2. Materials and Methods

### 2.1. Animals

As AD models, eight-month-old APP/PS1 double-transgenic mice were employed. This animal encodes a number of human AD genes, exhibits common clinical symptoms of AD, and is widely acknowledged in the pathophysiology of cognitive impairment [39, 40]. Because it is more precise, trustworthy, and effective, the transgenic AD mouse model is commonly utilized to replace the classic AD model [41]. Furthermore, at 7-8 months of age, these mice showed brain A*β* deposition [42, 43] and loss of local neurons [44], as well as learning and memory problems [45]. Shanghai Model Organisms provided eight-month-old APP/PS1 double-transgenic male mice. (Certificate number: SCXK (Ji) 2019-0008). The APP/PS1 mice (weighing 30 ± 2 g) were randomly divided into three groups: model (M), acupuncture (A), and memantine (ME), each with eight mice. The normal control (C) group consisted of six C57BL/6 male mice. To reduce external interference, mice were housed separately in standard mouse cages under constant temperature (23 ± 2°C) and constant humidity (40%-60%), with free access to water and food. The study was conducted in strict accordance with the regulations of the Animal Ethics Committee (20200811-01). Throughout the experiment, we made every effort to minimize animal suffering.

RETRACTED

### 2.2. Acupuncture Treatment

For a period of four weeks, the mice in acupuncture treatment group received acupuncture treatment for 20 minutes per day, five days per week, with two days off. Acupuncture points prescribed included Baihui (DU20), Hegu (LI4), Feishu (BL13), Pishu (BL20), Shenshu (BL23), Zusanli (ST36), and Sanyinjiao (SP6), as shown in Figure 1. The needles (diameter, 0.3 mm, Huatuo acupuncture of Suzhou Co., Ltd., Suzhou China) were inserted at a specific depth into corresponding acupoints.

### 2.3. Morris Water Maze (MWM) Test

After four weeks of acupuncture treatment, the mice's spatial learning and memory capacities were tested using the MWM test, as previously described [46]. The MWM device consists of a black circular tank (120 cm in diameter) filled with water (temperature 22-24°C) and a platform (12 cm in diameter) located 1 cm below the water surface in the platform quadrant. Mice were randomly assigned to one of the four quadrants facing the maze wall, where they can find a platform. If the platform was not discovered within 60 seconds, it would be directed there for 10 seconds. Mice were trained for four days which were used to examine spatial learning abilities and placed in three quadrants with no target platform. The escape latency, the distance to the target platform, and the swimming trajectories were recorded. The probe trail test was used to examine spatial memory abilities on the fifth day, and the platform was removed [46]. The mice were allowed to swim freely in water without a platform for 60 seconds. After this, the escape latency, the frequency of crossing the platform location, and the time spent on the platform quadrant were recorded.

### 2.4. Enzyme-Linked Immunosorbent Assay (ELISA)

Following the procedure, the blood obtained from decapitated mice was transferred to anticoagulant test tubes. After 2 hours at room temperature, the blood samples were centrifuged at 1000 rpm for 20 minutes, then we collected serum, and measured the levels of interleukin 1 beta (IL-1*β*) (ELISA Kit H002, Nanjing Jiancheng Bioengineering Institute), interleukin 10 (IL-10) (ELISA Kit H009, Nanjing Jiancheng Bioengineering Institute), lipopolysaccharides (LPS) (ELISA Kit A-054-2-1, Nanjing Jiancheng Bioengineering Institute), and tumor necrosis factor alpha (TNF-*α*) (ELISA Kit H052, Nanjing Jiancheng Bioengineering Institute) using an ELISA kit according to the manufacturer's instructions.

RETRACTED

### 2.5. Western Blot Analysis

Western blot(WB) was used to detect beta-amyloid 1-42 (A*β*) deposits and tau proteins expression in brain tissue samples. With a few exceptions, WB analysis was performed in accordance with conventional methods [47]. In brief, RIPA Lysis Buffer was used to lyse the total protein from each mouse hippocampal tissue sample, as directed by the manufacturer (Beyotime Institute of Biotechnology). The Bradford technique was used to determine the protein concentration. SDS-PAGE (8, 12, or 15% gel) was used to separate 20 g of protein, which was then transferred to the PVDF membrane. After 2 hours of blocking at room temperature with 5% skimmed milk, the membrane was incubated with particular primary antibodies overnight at 4°C. The primary antibodies utilized in this work were anti-beta-actin antibody (cat no. 25524-2-AP; 1 : 1000, Proteintech Group, Inc.) and anti-tau antibody (cat no. 66499-1-lg; 1: 10000; Proteintech Group, Inc.). The secondary antibody from the same genus was incubated at room temperature for 1.5 hours. Improved chemiluminescence detection reagent was used to improve imprinting detection (Beyotime Institute of Biotechnology). Image lab software can be used to evaluate and analyze band strength (Media Cybernetics, Inc., Rockville, MD, USA). The quantitative results were reported as a ratio of A*β* to *β*-actin and tau to *β*-actin and compared within each group to determine the relative changes.

### 2.6. DNA Extraction and 16SrDNA Gene Sequencing

The intestinal contents of mice were collected in a single sterile EP tube and immediately frozen at 80°C until DNA extraction was performed. The chloroform phenol DNA extraction method was used to extract the DNA from fecal samples. Thermo Nanodrop 2000 was used to determine the concentration of extracted DNA, and agarose gel electrophoresis was used to determine the molecular size. The V3-V4 region was then targeted using polymerase chain reaction amplification and 16SrDNA gene pyrosequencing. The Illumina Miseq platform was used to sequence the amplicon sequencing library, and the paired end read was 250 bp. The differences of bacterial abundance and diversity among different groups were analyzed by the Venn diagram, alpha diversity index, principal component analysis (PCA) et,al., and so on in order to study the bacterial differences among groups at each classification level, ANOVA analysis of variance was used.

### 2.7. Microbial Function Analysis

Using the 16SrDNA gene database, Phylogenetic Investigation of Communities by Reconstruction of Unobserved States (PICRUSt) of the community was carried out by reconstructing the unobserved state to predict the functional composition of the microbial community [48]. The related predicted genes and their functions were compared with the Kyoto Encyclopedia of Genes and Genomes (KEGG) database [49], and the differences between groups were compared using the STAMP software [50].

RETRACTED

### 2.8. Metabolomics Analysis

Metabolomics analysis was performed with liquid Chromatography-Quadrupole time of flight-mass spectrometry (LC-QTOF-MS, Waters, Shanghai, China) using an untargeted approach. Mouse feces samples (50 mg) were extracted with 80% methanol (800 *μ*L). The extract was sonicated for 30 minutes at 4°C, and centrifuged for 15 minutes at 4°C, 12000 rpm, and then removed for 200 *μ*L supernatant sparing. Chromatographic separations were performed on an Acquity HSS T3 column (2.1 × 1.8 *μ*m, Waters, Mississauga, ON, Canada) using a gradient programming of MS-grade water containing 0.05 percent formic acid (A) and acetonitrile (B). The mobile phase flow rate was 0.3 mL/min, the column temperature was 40°C, the injection volume was 3 *μ*L, and the temperature of the automated sampler was 4°C, the procedure is shown in Table 1. The eluted metabolites were analyzed in both positive and negative electrospray ionization mode with a full-scan ranging from 70 to 1050 m/z. All the raw files were first converted to mzML files by the ProteoWizard version 3.0 (Pala Alto, CA, USA), and data was processed for peak detection, retention time correction, alignment, and molecular feature annotation using the XCMS online version 3.7.1.

### 2.9. Statistics Analysis

The mean and standard deviation were used to represent the data. The SPSS 20.0 was used for statistical analysis, which included one-way ANOVA and the Student's *t*-test. A statistically significant difference was defined as *p* < 0.05.

PCA and Partial least squares-discriminant analysis (PLS-DA) were used to discriminate among the identified microbial metabolites using the tools provided in the MetaboAnalyst 5.0. The PLS-DA model was validated using cross-validation in order to avoid overfitting of the model. Variable Importance in the Project (VIP) scores based on the PLS-DA analysis were used to indicate the metabolites which significantly contributed to group separation. Pathway analysis tool provided in the MetaboAnalyst 5.0 was used to study the KEGG pathways among metabolites with VIP scores > 1.2.

## 3. Results

### 3.1. Acupuncture's Effect on the Spatial Learning Abilities of APP/PS1 Mice

MWM was used to test the spatial memory ability of the APP/PS1 mice. The spatial learning ability study was administered during the first four days of behavioral tests in the MWM. The mice struggled to find the platform on the first day of training, but by the fourth day, they were able to find the platform quickly (Figure 2(a)). The mice in the control group and acupuncture treatment group took the shortest path to the platform, while the path in the APP/PS1 model group was the longest and most complicated (Figure 2(a)). The escape latency of mice in each group decreased as training time increased (Figure 2(b)), and the distance to find the platform was reduced (Figure 2(c)), but there was no significant change in the average speed of platform searching (Figure 2(d)). The escape latency time of mice in each group was significantly reduced on the third day of training, indicating that mice in each group had essentially learned to find hidden platforms after three days of training. Interestingly, on the third and fourth day of training, acupuncture therapy reduced the mouse escape latency to the platform, bringing it closest to the control group. These data suggested that acupuncture could have a beneficial effect on the spatial learning capacity of the APP/PS1 mice.

RETRACTED

### 3.2. Acupuncture's Effect on the Spatial Memory Abilities of APP/PS1 Mice

MWM test was performed on the fifth day to investigate the effect of acupuncture on spatial memory ability of the APP/PS1 mice. When the platform was removed, the mice's escape latency to the platform quadrant (Figure 2(e)), the average speed (Figure 2(f)), the quadrant frequency (Figure 2(g)), and the percentage of time spending in the platform quadrant were tested (Figure 2(h)). The escape latency of the APP/PS1 model group was the longest, which was significantly higher than that of the control group (*p* <0.05). The escape latency of acupuncture treatment group did not vary significantly from the APP/PS1 model group and control group, respectively. However, the escape latency of acupuncture treatment group was closer to that of the control group (Figure 2(e)), suggesting that acupuncture could shorten the escape latency of the APP/PS1 mice. In addition, as shown in Figures 2(f)–2(h), the average speed, frequency of passing through the target quadrant, and percentage of time spent in the platform quadrant all showed highly similar results as compared to the results of escape latency. Since the acupuncture treatment mice received more information in the spatial learning training, more memory could be retrieved in this test [51], causing the acupuncture treatment group's parameters to tend to the level of the control group. Moreover, the acupuncture treatment group's therapeutic outcome was also quite close to that of the positive control group. These data suggested that acupuncture could have a beneficial effect on the spatial memory capacity of APP/PS1 mice.

RETRACTED

### 3.3. Acupuncture May Regulate A*β* and Tau Protein Expression in the Hippocampus of APP/PS1 Mice

The accumulation of A*β* in the brain is thought to be the main feature of AD [24]. Amyloid plaques in the hippocampus can cause neuronal loss and cognitive dysfunction [21, 25]. The effect of acupuncture on A*β* deposition was investigated further in this research. WB analysis showed that the amount of A*β* in the APP/PS1 model group's hippocampus tissue increased, and acupuncture treatment was able to reduce this increase significantly (*p* < 0.05, Figures 3(a) and 3(b)). Tau protein accumulation and the presence of neurofibrillary tangles were more closely related to symptom severity and neuron death in humans than A*β* lesions [51]. According to our findings, the acupuncture treatment group's expression of tau protein in the hippocampus was lower as compared to the model group, but there was no substantial difference between the two groups. In addition, the acupuncture treatment group's therapeutic effects on the expression of A*β* and Tau protein were also similar to that of the positive control group. These findings suggested that acupuncture could regulate the expression of A*β* and tau protein in the APP/PS1 mice.

### 3.4. Acupuncture Regulates Inflammatory Factors in APP/PS1 Mice

Many findings suggested that neuroinflammation plays a key role in the development of the neuropathological changes seen in AD [52]. In our research, ELISA was used to detect the expressions of IL-1*β*, IL-10, LPS, and TNF-*α* in the mice's serum (Figures 4(a)–4(d)). Our findings indicated that there was no significant difference in the IL-10 expression between the control and model groups, but the IL-10 expression of the model group's rose in comparison to the control group. Meanwhile, when compared to the model group, the positive control group and acupuncture treatment group had significantly lower IL-10 levels (*p* < 0.01, Figure 4(a)), showing that acupuncture may have a regulatory influence on the level of IL-10 in the APP/PS1 mice. In addition, acupuncture treatment reduced LPS in the mice's serum significantly (*p* < 0.05, Figure 4(c)). However, there was no significant difference in IL-1*β* and TNF-*α* expression among the four groups (Figures 4(b) and 4(d)).

### 3.5. Acupuncture Regulates the Gut Microbiota of APP/PS1 Mice

Since the aforementioned studies had demonstrated that the therapeutic effect of acupuncture was close to that of positive drug, however, the primary goal of this research was the effect of acupuncture, we excluded the positive drug group from the gut microbiota and metabolites research and studied the gut microbiota composition among the control group, APP/PS1 model group, and acupuncture treatment group in this section.

RETRACTED

We used 16srDNA detection on the feces of the mice to investigate the impact of acupuncture on the gut microbiota. A total of 672 operational taxonomic units (OTUs) were displayed at a 97 percent similarity level. The Venn diagram revealed that the three groups shared 327 OTUs, with 85 OTUs unique to the control group, 40 OTUs unique to the APP/PS1 model group, and 30 OTUs unique to the acupuncture treatment group (Figure 5(a)). On the rarefaction curve, the number of organisms observed increased as the amount of sequencing data increased. When a certain amount of sequencing data was reached, the rarefaction curve exhibited a relatively stable condition, suggesting that the amount of sequencing data of samples was reasonable (Figure 5(b)). According to the Shannon and Simpson indices (Figures 5(c) and 5(d)), the APP/PS1 mice had lower gut microbiota diversity, and acupuncture appeared to regulate gut microbiota diversity; however there was no statistical difference (*p* > 0.05).  Figure 6 illustrates the phylum-level variations and relative abundance of the three groups. Bacteroidetes and Firmicutes had the highest relative abundance of the three groups (Figure 6(a)). The APP/PS1 model group and acupuncture treatment group varied greatly from the control group, and there was no statistically significant difference between the model and acupuncture treatment groups (Figure 6(b)). Actinobacteria varied among the three groups. The APP/PS1 model group varied substantially from the control and acupuncture treatment groups (*p* < 0.05), but there was no difference between the control and acupuncture treatment groups (Figure 6(b)). To explore the differences in gut microbiota among the three groups further, we performed PCA analysis of the microbiota of each group to visualize the differences.  Figure 6(c) demonstrates the PCA results as a score graph. The variance of the two principal components (axis 1 and axis 2) in the mouse OTU data was found to account for 51.942 percent and 17.357 percent of the overall variance, respectively. The results revealed three independent clusters clearly among groups.

Following that, we used the LDA Effect Size (LEfSe) analysis on the I-Sanger platform to classify the communities in the study. LEfSe can be compared across several classes to classify bacterial species with major abundance differences.  Figure 7 depicts the differences in the bacterial taxa of mice among the three groups. The diameter of the circle represented the species' abundance. The radial circles reflected the classification level from phylum to species, from inside to outside (phylum-class-order-family-genus-species). A classification was defined by each small circle on a different classification stage. The small circle's diameter was proportional to its relative abundance. The degree of species annotation was defined by the fan-shaped region drawn from the inside to the outside. The color of the gut microbiota varies, and species that were not distinct had to be colored yellow. The red node represented a microbial group that was important in the control group, the green node represented a microbial group that was important in the APP/PS1 model group, and the blue node represented a microbial group that was important in the acupuncture treatment group. The cladogram revealed 62 taxa (9 classes, 9 orders, 19 families, and 25 genera) that differed in abundance among the three groups.  Figure 8 depicts the LDA scores of the three groups with major differences, which were determined by selecting the top ten species in each group with the lowest *p* value from the LEfSe results. The length of the bar graph reflected the contribution of individual bacteria for the classification among different groups.

RETRACTED

Next, we explored the gut microbiota variations among the three groups at the family stage.  Figure 9(a) depicts the top 24 bacterial families in each of the three groups in terms of relative abundance. There were ten bacterial families with statistically important variations (*p* < 0.05), and the four dominant bacterial families in the three groups were Porphyromonadaceae, Lactobacillaceae, Bacteroidaceae, and Prevotellaceae (Figures 9(b) and 9(c)). Acupuncture treatment significantly changed the relative abundance of ten families, and the abundance of nine bacteria families tended to be similar to the control group (Figures 9(b) and 9(c)). In addition, acupuncture therapy reduced significantly the relative abundance of Porphyromonadaceae (*p* < 0.05), Coriobacteriaceae (*p* < 0.05), Helicobacteraceae (*p* < 0.05), and Burkholderiaceae (*p* < 0.01) of the APP/PS1 mice (Figure 9(b)). Moreover, acupuncture treatment was able to increase significantly the relative abundance of Christensenellaceae (*p* < 0.01), Clostridiaceae 1 (*p* < 0.01), Prevotellaceae (*p* < 0.05), Rikenellaceae (*p* < 0.05), and Bacteroidaceae (*p* < 0.05) of the APP/PS1 mice (Figure 9(c)). Furthermore, there was a statistically significant difference in Lactobacillaceae between the APP/PS1 model and control group (*p* < 0.001). The difference was more distinct between the acupuncture treatment and control group (*p* < 0.0001). The relative abundance of Lactobacillaceae was able to increase by acupuncture, indicating an inverse tendency compared to the control group.

RETRACTED

Following that, we used PICRUSt to examine and predict the functional gene composition in the metabolic pathway. To identify the functional genes with significant differences, ANOVA was used to compare the relative abundance of functional genes among the three classes. The screening threshold for substantial differences was set at *p* < 0.05. The metabolic pathway prediction was created for functional genes with large differences in relative abundance among the three groups. Supplementary Figure S1 depicts the effects.

### 3.6. Acupuncture Regulates the Microbial Metabolites of APP/PS1 Mice

A total of 697 metabolites were detected in the fecal extract samples after peak filtering and blank subtraction. Multivariate statistical analyses were carried out using the MetaboAnalyst 5.0 to reveal the changes in metabolite among groups in the 697 compounds results. The variations in metabolic profiles between the control group, model group, and acupuncture group were originally visualized by PCA (Figure 10(a)) but no important clusters among the three groups were found in PCA analysis. A supervised clustering method—PLS-DA—had therefore been carried out for optimal separation and identifying the components that significantly contribute to the division. The PLS-DA assessment showed the major variations between the classes with 0.86 predictive accuracy and 0.96 goodness-of-fit (R2) among the three groups (Figure 10(b)). The classification was based on 99 metabolites with VIP scores of >1.2 (Table 2). Table 2 lists the up and downregulation patterns among the three groups of these metabolites. The metabolic pathway study was conducted using the MetaboAnalyst 5.0, based on the KEGG data of these metabolites, shown in Table 2. The findings revealed that the most important metabolic pathways relating to the regulation effect of acupuncture were pyrimidine metabolism; alanine, aspartate, and glutamate metabolism; arginine biosynthesis; phenylalanine, tyrosine, and tryptophan biosynthesis; linoleic acid metabolism; D-glutamine and D-glutamate metabolism; taurine and hypotaurine metabolism and phenylalanine metabolism (Figure 11), and six of these pathways were consistent with the PICRUSt analysis prediction (Supplementary Figure S1), except alanine, aspartate, and glutamate metabolism and aginine biosynthesis.

## 4. Discussion

According to traditional Chinese medicine (TCM) theory, the pathogenesis of AD is closely related to internal organ insufficiency. Qi is the energy that sustains the life system based on the principle of TCM. Qi circulates in specific meridians of the body, and a blockage of Qi circulation will result in organ dysfunction. As a result, acupoints in particular meridians are often chosen to treat illness. The Governor meridian has the ability to collect Qi and facilitate Qi circulation through the brain. The Bladder Meridian runs through the brain. Therefore, Baihui acupoints above the Governor meridian; Feishu, Pishu, and Shenshu on the Bladder meridian were used to treat the APP/PS1 mice. Since recent research has linked gut microbiota to AD, Sanyinjiao, Zusanli, and Hegu acupoints on the digestive system related meridians were chosen. Our results indicate that stimulating these acupoints simultaneously has a positive impact on the cognitive ability of the APP/PS1 mice. This result agrees with previous studies [39, 40].

RETRACTED

In the MWM study, the performance of mice in the MWM hidden platform training and probe tests after four weeks of acupuncture was comparable to that of the control group, indicating that acupuncture could have a beneficial effect on the spatial learning and memory capacities of the APP/PS1 mice, which is consistent with previous findings [39–41, 46] using AD animal models. In the test of spatial learning capacity based on MWM, the escape latency (Figure 2(b)) and travelled distance (Figure 2(c)) in each group dropped dramatically as learning time increased, demonstrating that after four days of training, each group's animals had a basic comprehension of the spatial distribution of the water maze. However, the parameter speed (Figure 2(d)) did not reveal such a time-dependent variation. Three groups of animals, excluding the control group, had a reduced swimming speed on the fourth day of training. This could be because the animals are unfamiliar with the maze's spatial structure during the first three days of training. Through rapid swimming behavior, animals learned how to select the optimal way, resulting in a longer escape time and traveling distance. However, on the fourth day, even if the animals' swimming speed was decreased, they could rapidly exit the maze via the optimal way. At this point, the slow swimming speed may be explained by the animals having adapted to the water maze's surroundings and comprehending the maze's spatial structure. There is no reason to increase one's swimming speed and attempt the maze's exit repeatedly. On the other hand, the animals who demonstrated a decreased speed on the third day of training were the C57BL/6 mice, which may be a strain-specific tendency. The more particular mechanism underlying this behavior warrants additional investigation. In the test of spatial memory capacity based on MWM, all parameter values in the acupuncture treatment group were comparable to those in the control group, with no significant difference, indicating that acupuncture had a positive regulatory effect on the memory ability of the APP/PS1 mice.

RETRACTED

A*β* plaque and tau protein-containing neurofibrillary tangles are two neuropathological features of AD that are believed to play a role in the neurodegenerative pathway that leads to dementia [53]. A*β* is the main component of senile plaques and a typical pathway product of AD [54], and its overproduction or accumulation is critical to the pathogenesis of AD [55]. Although numerous research on phosphorylated tau (p-tau) alterations in the APP/PS1 mice have been conducted in the past, while the AD Association's working group considers the total tau (t-tau) and p-tau to be equivalent in determining the disease's status [56]. As a result, we focused on t-tau changes in our study, which is compatible with the guidelines developed by the AD Association's work group on AD diagnosis. Tau protein production occurs prior to the onset of degeneration, implying that tau protein is the primary cause of AD neurodegeneration. Acupuncture can reduce the expression of A*β* and tau proteins in the hippocampus, suggesting that the molecular basis of acupuncture in the treatment of AD.

IL-10 is an anti-inflammatory cytokine found in healthy brain tissue, but it is overexpressed in AD patients [57]. IL-10 can promote neuroinflammation and microglia dysfunction, resulting in reducing A*β* clearance, increasing A*β* burden, and cognitive decline [58]. The brains of the IL-10-deficient APP/PS1 mice had a higher number of activated microglia, as well as improved A*β* clearance, reduced A*β* accumulation, and declined modest cognition [59, 60]. Several investigations based on genome-wide association analyses supported our findings, which also showed that IL-10 was increased in the brain of AD [61, 62]. Acupuncture dramatically decreases IL-10 in the APP/PS1 mice, which may reduce A*β* deposition and improve learning and memory.

LPS, as a unique component of Gram-negative bacteria's outer membrane, is vital in host-pathogen interactions and the innate immune system [63]. LPS is strongly proinflammatory to human neurons, resulting in the production of proinflammatory signals [64], an increase in A*β* [65, 66], and Tau hyperphosphorylation [67, 68]. LPS was identified in significant amounts in the neocortex and hippocampus of the brain during AD [69]. More and more data indicates that LPS can enter the systemic circulation via the portal vein and subsequently affected brain tissue, which is a key source of inflammatory deterioration in AD [70]. Our findings revealed that LPS levels in the APP/PS1 model group's blood were significantly raised and that they might be greatly reduced by acupuncture. This corresponded to prior research findings that acupuncture at Zusanli had been demonstrated to stimulate anti-inflammatory pathways and drastically lower proinflammatory cytokines [71]. Based on the findings, acupuncture may reduce A*β* deposition and tau phosphorylation by lowering LPS levels, and so have a therapeutic effect on AD.

RETRACTED

Acupuncture has been explored in recent years to improve gut microbiota [36, 37], signaling that the gut microbiota could be a suitable target for the therapeutic effect of acupuncture. Atypical gut microbiota has been observed in some AD investigations [20–27]. As a result, we focused on the changes in the gut microbiota of AD model mice. According to our research, the gut microbiota of the APP/PS1 mice changed dramatically. The gut ecology of the APP/PS1 mice had been demonstrated to be altered by acupuncture. The APP/PS1 mice had a lower diversity of gut microbiota, but acupuncture appeared to boost gut microbiota diversity (Figure 5). The concentration of germs on phylum and family levels was comparable in the acupuncture treatment group and APP/PS1 model group. At the phylum level, Bacteroides and Firmicutes had the highest relative abundance. The model group had the largest relative abundance of Actinobacteria, which differs significantly from the control and acupuncture treatment groups (Figure 6). Previous research revealed an increase in the relative abundance of Actinobacteria in the feces of the APP/PS1 mice and AD patients [72–74]. Actinobacteria secretes chemotactic and proinflammatory cytokine-inducing proteins, activates complement pathways, and generates hyaluronidases, proteases, and neuraminidases, all of which are expected to induce epithelial permeabilization and inflammatory infiltration [75]; therefore, Actinobacteria may contribute to the advancement of AD. According to our findings, acupuncture may have a therapeutic effect on AD by lowering abundance of Actinobacteria.

At the family level, the relative abundance of Porphyromonadaceae [76] and Helicobacteraceae [77] was shown to be quite high in the APP/PS1 mice, which was consistent with earlier findings. Many Porphyromonadaceae species are part of the indigenous microbiota of the human and animal gastrointestinal tract and oral cavity; however, some have been linked to a variety of human and animal infections [78]. The increased Helicobacteraceae expression was primarily owing to the increased Helicobacter. Infection with pathogenic microorganisms such as Helicobacter pylori can worsen A*β* development and Tau phosphorylation, increasing the likelihood of AD [79, 80]. Acupuncture dramatically reduced the amount of Porphyromonadaceae and Helicobacteraceae in this study, indicating that the gut microbiota components impacted by acupuncture may interfere with AD.

RETRACTED

In this study, we also discovered that the quantity of Bacteroidaceae was low in the APP/PS1 mice, which was consistent with earlier findings [73, 81]. Bacteroidaceae expression declined predominantly as a result of a fall in Bacteroides quantity. Previous research found low levels of Bacteroidaceae in patients with cognitive impairment and brain amyloidosis [82]. Acupuncture significantly increased the amount of Bacteroidaceae in this study, showing that acupuncture may have a therapeutic effect on AD by altering intestinal flora.

Acupuncture increased the expression of Lactobacillaceae to some level in this study. Lactobacillaceae overgrowth has already been documented in the APP/PS1 mice [83, 84]. Lactobacillaceae is a Firmicutes phylum family of Gram-positive, non-spore-forming, fermentative bacteria that are generally thought to be helpful to humans. The main reason for the increase in Lactobacillaceae in this study was an increase in Lactobacillus relative abundance. Lactobacillus has been found in AD rats to improve memory and learning problems [85]. Simultaneously, human investigations have revealed that the concentration of Lactobacillus is related to age [86]. These data imply that Lactobacillus plays an important role in the development of AD. According to Wang et al., Lactobacillus may improve cognitive impairment caused by prolonged stress in rats [87]. Lactobacillus fermentum NS9 treatment increased memory ability [88].

Metabolites produced by host and intestinal bacteria exert important and diverse effects on various diseases including AD [89]. Acupuncture modified a huge number of metabolites in the APP/PS1 mice's feces, according to our findings. The VIP score was used to investigate the altered metabolites, and then, the KEGG metabolic pathway was examined. PICRUSt study targeting the quantity of gut microbiota discovered six metabolic pathways that were compatible with the KEGG pathway predicted results. These six pathways have been linked to the occurrence, development, and treatment of neurodegenerative disorders in previous studies [90–94]. This shows that acupuncture-induced changes in gut flora and metabolites may alter the learning and memory abilities of the APP/PS1 mice in this research. It is important to remember that acupuncture is a holistic and systemic treatment. Acupuncture has the ability to influence not only the number of intestinal microorganisms but also metabolites, allowing it to govern the biological system as a whole. As a result, when paired with intestinal flora and metabolites to research the effect of acupuncture, the intervention effect of acupuncture on AD may be revealed more fully. However, in this study, we employed nontargeted metabolomics technology to detect metabolites, which on the one hand extended the types of metabolites, but on the other hand rendered our metabolites insufficient to focus on specific metabolic pathways, such as the bile acid metabolic pathway. Future research could look at employing a targeted metabolomics platform to explore specific metabolite pathways in order to give more reliable biological evidence for the effect of acupuncture intervention on AD.

RETRACTED

## 5. Conclusions

In this study, acupuncture was demonstrated to improve the learning and memory ability of the APP/PS1 mice. Acupuncture may lower A*β* deposition and t-tau protein content in the brain hippocampus of the APP/PS1 mice, control inflammatory factor release, and alter intestinal flora and metabolites. Therefore, acupuncture, as a holistic therapy, has the potential to significantly contribute in the treatment and control of AD. Gut dysregulation and intestinal microbial-host interaction now play a major role in neurodegenerative illness, according to growing experimental and clinical evidence. While several promising biomarkers were discovered in our study, more research into how to use these biomarkers to examine the therapeutic effects of acupuncture on AD are required. Methods of changing the composition of the microbiome through acupuncture require further research. In conclusion, this study adds to our understanding of the effect of acupuncture on AD and opens the door to further research into the alterations of intestinal bacteria in the presence of AD.

## Figures and Tables

**Figure 1:** Schematic diagram of acupuncture points on the mouse body. DU20 was only one acupoint. LI4, BL13, BL20, BL23, ST36, and SP6 were symmetrical on both sides of the body. DU20 is located in the middle of parietal bone; LI4 is located between the first and second metacarpal bones of the forelimb; BL13 is located on bilateral intercostal area, just below the third thoracic vertebra; BL20 is located on bilateral intercostal area, just below the 11th thoracic vertebra; BL23 is located on bilateral intercostal area, just below the second lumbar vertebra; ST36 is located at the posterolateral side of the knee joint, about 2 mm below the small head of fibula; and SP6 is located about 5 mm above the straight point of the inner ankle of the hind limb.

RETRACTED

**Figure 2:** Acupuncture improves APP/PS1 mice's learning and memory abilities on day 1 to day 4 (a–d) and the day 5 (e–h) of the MWM test, respectively. (a) The training traces of each group on the first and fourth day. (b) A comparison of each group's escape latency from day 1 to day 4. (c) A comparison of each group's distance from day 1 to day 4. (d) A comparison of each group's average speed from day 1 to day 4. (e) A comparison of each group's escape latency on the fifth day. (f) A comparison of each group's average speed on the fifth day. (g) A comparison of each group's passing times through the platform quadrant on the fifth day. (h) A comparison of each group's percentage of elapsed time through the platform quadrant on the fifth day. ^∗^*p* < 0.05.

**Figure 3:** WB analysis of the effects of acupuncture treatment on hippocampal A*β* and Tau expression levels in the APP/PS1 mice. (a) A strip of Western blotting paper. C: control group; M: APP/PS1 model group; A: acupuncture treatment group; ME: memantine group. (b) Quantitative assessment of A*β* expression levels in the hippocampus. (c) Quantitative evaluation of tau protein expression levels in the hippocampus.

**Figure 4:** Effects of acupuncture treatment on the expression of IL-10, IL-1*β*, LPS, and TNF-*α* in mice's serum samples using ELISA. ^∗^*p* < 0.05; ^∗∗^*p* < 0.01.

**Figure 5:** Evaluation of sequencing data from the mice's fecal samples. (a) Venn diagram showed the number of OTUs in the three groups. C: control group; M: APP/PS1 model group; A: acupuncture treatment group. (b) Rarefaction curves indicate whether the amount of sequencing data of the sample is reasonable. C: control group; M: APP/PS1 model group; A: acupuncture treatment group. (c) Shannon index revealed that *α*-diversity and richness are intertwined. (d) Simpson index showed the variety, which included both *α*-diversity and richness.

**Figure 6:** Microbial composition structures at the phylum level of mice in the three groups. (a) Amounts of relative abundance (%) of bacterial taxa at the phylum level. (b) Significantly different bacterial taxa at the phylum level of mice in the three groups. ^∗^*p* < 0.05; ^∗∗^*p* < 0.01. (c) PCA results of beta diversity calculated of mice's OTU data among the three groups. C: control group; M: APP/PS1 model group; A: acupuncture treatment group.

**Figure 7:** Cladograms generated by LEfSe indicating differences in the bacterial taxa of mice among the three groups. C: control group; M: APP/PS1 model group; A: acupuncture treatment group.

**Figure 8:** LDA scores for the differentially abundant bacterial taxa among the three groups. LDA scores > 2.0 are shown. C: control group; M: APP/PS1 model group; A: acupuncture treatment group.

RETRACTED

**Figure 9:** Microbial community structures at the family level of mice, and the different groups had substantially different bacterial taxa at the family level. ^∗^*p* < 0.05, ^∗∗^*p* < 0.01, ^∗∗∗^*p* < 0.001, ^∗∗∗∗^*p* < 0.0001.

**Figure 10:** PCA and PLS-DA scores obtained from the metabolites data. (a) PCA and (b) PLS-DA score plots of the metabolites data obtained from identified compounds.

**Figure 11:** Bubble plots showing the altered metabolic pathways in mice.

**Table 1:** Procedure for gradient elution in the mobile phase.

Time (min)	Flow rate (mL/min)	*A* (%)	*B* (%)
0	0.3	95	5
1	0.3	95	5
12	0.3	5	95
13.5	0.3	5	95
13.6	0.3	95	5
16	0.3	95	5

**Table 2:** List of relevant metabolites identified by VIP scores.

No	Compound	VIP scores	KEGG	M vs. C	A vs. M
1	2-Hydroxymyristic acid	2.3674	NA	↑^∗∗∗^	↓^∗∗∗^
2	Cortisol	2.2876	C00735	↓^∗∗^	↑^∗∗∗^
3	Costunolide	2.1317	NA	↓^∗^	↑^∗∗∗^
4	5-Fluorouridine	2.0918	C16633	↑^∗∗^	↓^∗∗∗^
5	Benzyl cinnamate	1.9261	NA	↑^∗^	↓^∗∗^
6	6-Hydroxymelatonin	1.9253	C05643	↑	↓^∗∗∗^
7	Cymarin	1.9074	NA	↑	↓^∗∗∗^
8	Pravastatin	1.858	C01844	↑^∗∗^	↓^∗∗^
9	Ascorbic acid	1.8468	C01041	↑	↓^∗∗^
10	Crotonic acid	1.8403	C01771	↓	↑^∗∗^
11	Testosterone enanthate	1.8348	C08157	↑^∗^	↓^∗∗^
12	D-Serine	1.8304	C00740	↓	↑^∗∗^
13	Gly-Tyr	1.8304	NA	↑	↓^∗∗∗^
14	Cholic acid	1.8283	C00695	↑^∗^	↓^∗∗^
15	Deoxycholic acid	1.8261	C04483	↑^∗^	↓^∗∗^
16	Cotinine	1.8094	NA	↑	↓^∗∗∗^
17	L-Methionine sulfoxide	1.7992	NA	↑^∗∗^	↓^∗∗^
18	Acetyl tributyl citrate	1.7963	NA	↓	↑^∗∗^
19	Asiatic acid	1.7772	NA	↑^∗^	↓^∗∗^
20	L(+)-Ornithine	1.7701	NA	↑	↓^∗∗∗^
21	Gallic acid	1.7472	C01424	↑^∗^	↓^∗∗^
22	Mephobarbital	1.74	C07829	↑^∗∗∗^	↓^∗∗^
23	Taurine	1.7381	C00245	↑	↓^∗∗^
24	Deoxyuridine	1.7271	C00526	↑^∗^	↓^∗∗^
25	5*α*-Dihydrotestosterone	1.7155	NA	↑^∗∗^	↓^∗∗^
26	Propionylcarnitine	1.7107	C03017	↑	↓^∗∗^
27	N6,N6,N6-Trimethyl-L-lysine	1.7059	C03793	↓	↑^∗∗^
28	Tributyl phosphate	1.6935	NA	↓^∗^	↑^∗∗^
29	Desthiobiotin	1.6798	C01909	↑^∗∗^	↓^∗∗^
30	Prolylyphenylalanine	1.6725	NA	↑^∗∗∗^	↓^∗∗^
31	Jasmonic acid	1.6723	C08491	↓^∗^	↑^∗∗^
32	Glycodeoxycholic acid	1.6494	C05464	↑	↓^∗∗^
33	N-Formylmethionine	1.6231	NA	↑	↓^∗^
34	Thymine	1.6229	C00178	↑^∗∗^	↓^∗∗^
35	Genistein 4'-O-glucuronide	1.6162	NA	↑	↓^∗∗^
36	Glu-Val-Phe	1.5995	NA	↑	↓^∗^
37	Meprobamate	1.5918	NA	↑	↓^∗∗^
38	herniarin	1.5889	C09268	↓	↑^∗∗^
39	Stearamide	1.5853	C13846	↓	↑^∗^
40	Uracil	1.5764	C00106	↑	↓^∗^
41	Kahweol	1.5601	NA	↓^∗^	↑^∗∗^
42	Linoleic acid	1.5531	C01595	↑^∗^	↓^∗^
43	Valylproline	1.5507	NA	↑^∗^	↓^∗∗^
44	D-Sphingosine	1.5441	NA	↑	↓^∗^
45	Eicosapentaenoic acid	1.5282	C06428	↑^∗∗^	↓^∗^
46	Alanyltyrosine	1.5281	NA	↑	↓^∗∗^
47	Monobutylphthalate	1.5274	NA	↓	↑^∗∗∗^
48	Hydroxyphenyllactic acid	1.5262	C01207	↑^∗^	↓^∗^
49	L-Phenylalanine	1.5259	C00079	↑^∗^	↓^∗^
50	L-Pyroglutamic acid	1.5225	C01879	↑	↑^∗∗^
51	Diisobutylphthalate	1.5224	NA	↓	↑^∗∗^
52	Taurodeoxycholic acid	1.5198	C05463	↓	↑^∗∗^
53	2-Methyl-S-benzothiazole	1.5025	NA	↓	↑^∗∗^
54	Coumarin	1.4947	C05851	↓^∗∗^	↑^∗^
55	Perillartine	1.4923	NA	↓	↑^∗∗^
56	Asiaticoside	1.4824	C15428	↑	↑^∗^
57	Oleanolic acid	1.4788	C17148	↑	↓^∗^
58	Nateglinide	1.4757	NA	↑	↓^∗^
59	DL-Glutamine	1.4374	C00303	↑	↑^∗^
60	N-Acetylaspartic acid	1.4348	C01042	↑^∗^	↓^∗^
61	N-Acetyl-L-leucine	1.433	C02710	↑	↓^∗^
62	Gluconolactone	1.4319	NA	↓	↑^∗^
63	5-Hydroxy-L-tryptophan	1.4087	NA	↓	↑^∗^
64	Limonene	1.4042	NA	↓	↑^∗^
65	Glu-Gln	1.394	NA	↓	↑^∗^
66	Dodecyl sulfate	1.392	C08031	↓^∗∗^	↑^∗^
67	Dihydrothymine	1.379	NA	↑	↓^∗^
68	Gabapentin	1.3722	D00332	↓	↑^∗^
69	Thiamine	1.3713	C00378	↓	↑^∗^
70	Arachidonic acid	1.3673	C00219	↑^∗∗^	↓^∗^
71	Alpha,alpha-Trehalose	1.3651	C01083	↑	↑^∗^
72	6-Methylquinoline	1.3557	NA	↑	↓^∗^
73	Daidzin	1.3546	C10216	↓	↑^∗^
74	Gly-Val	1.351	NA	↑	↓^∗^
75	N5-Acetylornithine	1.3466	NA	↑	↓^∗^
76	Benzothiazole	1.3405	NA	↑^∗^	↑^∗^
77	Uridine monophosphate (UMP)	1.328	C00105	↑	↓^∗∗^
78	L-Aspartic acid	1.3063	C00049	↓	↑^∗^
79	Crustecdysone	1.3018	NA	↓	↓^∗^
80	2,3,4,9-Tetrahydro-1H-beta-carboline-3-carboxylic acid	1.2957	NA	↓	↑^∗^
81	2,2,6,6-Tetramethyl-1-piperidinol (TEMPO)	1.2921	NA	↓	↑^∗^
82	Imazamox	1.2899	C18598	↑^∗^	↓^∗^
83	2,4-Quinolinediol	1.2814	C16716	↑	↓^∗^
84	5-Thymidylic acid	1.2799	C00364	↑^∗^	↓^∗^
85	Thymidine	1.2671	C00214	↑	↓^∗^
86	8-HETE	1.2615	C14776	↑	↓
87	N2,N2-Dimethylguanosine	1.2596	NA	↓^∗^	↑^∗^
88	p-Coumaraldehyde	1.257	NA	↓	↑^∗^
89	Pyridoxine	1.2569	NA	↓	↑^∗^
90	Glycyl-L-leucine	1.2534	C02155	↑	↓^∗^
91	L-Glutamic acid	1.2445	C00025	↓	↑
92	5-Hydroxytryptophan	1.2438	C01017	↓	↑^∗^
93	Neocnidilide	1.2399	NA	↑	↑
94	Isophorone	1.2268	C14743	↓	↑
95	6-Hydroxycaproic acid	1.2208	NA	↑	↑^∗^
96	Xanthosine	1.2103	C01762	↑	↓
97	Pentadecanoic acid	1.2077	C16537	↑^∗^	↓
98	Pachyrrhizin	1.2051	NA	↓^∗^	↑^∗^
99	Prolinamide	1.2024	C19781	↓	↑

The sequence of the metabolites indicates their importance for the contribution to the group separations. “↑” in M vs. C indicates that specific metabolites in the APP/PS1 model group are upregulated in comparison to the control group. “↓” in M vs. C indicates that specific metabolites in the APP/PS1 model group are downregulated in comparison the to control group. “↑” in A vs. M indicates that specific metabolites in the acupuncture treatment group are upregulated in comparison to the APP/PS1 model group. “↓” in A vs. M indicates that specific metabolites in the acupuncture treatment group are downregulated in comparison to the acupuncture treatment group. “^∗^” reveals the significant difference of metabolites abundance between the two groups determined by Student's *t*-test, ^∗∗∗^: *p* < 0.001: ^∗∗^: *p* < 0.01; ^∗^: *p* < 0.05.

RETRACTED

## Data Availability

The datasets generated during and/or analyzed during the current study are available from the corresponding author on reasonable request.

## Supplementary Materials

Supplementary Materials Figure S1: the supplementary material depicts the effects among different groups of microbiota data predicted by PICRUSt analysis.

## References

[1] Long J. M., Holtzman D. M. (2019). Alzheimer disease: an update on pathobiology and treatment strategies. *Cell*.

[2] Park S., Lee J. H., Yang E. J. (2017). Effects of acupuncture on Alzheimer's disease in animal-based research. *Evidence-Based Complementary and Alternative Medicine*.

[3] Arvanitakis Z., Shah R. C., Bennett D. A. (2019). Diagnosis and management of dementia: review. *JAMA*.

[4] Zhang F., Zhong R. J., Cheng C., Li S., Le W. D. (2021). New therapeutics beyond amyloid-*β* and tau for the treatment of Alzheimer's disease. *Acta Pharmacologica Sinica*.

[5] Szeto J. Y. Y., Lewis S. J. G. (2016). Current treatment options for Alzheimer's disease and Parkinson's disease dementia. *Current Neuropharmacology*.

[6] Livingston G., Sommerlad A., Orgeta V. (2017). Dementia prevention, intervention, and care. *Lancet*.

[7] Schwarz S., Froelich L., Burns A. (2012). Pharmacological treatment of dementia. *Psychiatry*.

[8] Desai A. K., Grossberg G. T. (2005). Diagnosis and treatment of Alzheimer’s disease. *Neurology*.

[9] Wang Z., Liang P., Zhao Z. (2014). Acupuncture modulates resting state hippocampal functional connectivity in Alzheimer disease. *PLoS One*.

[10] Takizawa C., Thompson P. L., Van Walsem A., Faure C., Maier W. C. (2015). Epidemiological and economic burden of Alzheimer's disease: a systematic literature review of data across Europe and the United States of America. *Journal of Alzheimer’s Disease*.

[11] Jung Y. J., Kim Y. H., Bhalla M., Lee S. B., Seo J. (2018). Genomics: new light on Alzheimer's disease research. *International Journal of Molecular Sciences*.

[12] Yu L., Petyuk V. A., Gaiteri C. (2018). Targeted brain proteomics uncover multiple pathways to Alzheimer's dementia. *Annals of Neurology*.

[13] Wilkins J. M., Trushina E. (2017). Application of metabolomics in Alzheimer's disease. *Frontiers in Neurology*.

[14] Chandra N., Srivastava A., Kumar S. (2019). Bacterial biofilms in human gastrointestinal tract: an intricate balance between health and inflammatory bowel diseases. *World Journal of Pharmacology*.

RETRACTED

[15] Ding R., Goh W., Wu R. (2019). Revisit gut microbiota and its impact on human health and disease. *Analysis*.

[16] Vila A. V., Imhann F., Collij V. (2018). Gut microbiota composition and functional changes in inflammatory bowel disease and irritable bowel syndrome. *Science Translational Medicine*.

[17] Frost F., Kacprowski T., Rühlemann M. (2019). Impaired exocrine pancreatic function associates with changes in intestinal microbiota composition and diversity. *Gastroenterology*.

[18] Kurilshikov A., van den Munckhof I. C. L., Chen L. (2019). Gut microbial associations to plasma metabolites linked to cardiovascular phenotypes and risk. *Circulation Research*.

[19] Neill C. O. (2019). Gut microbes metabolize Parkinson's disease drug. *Science*.

[20] Varesi A., Pierella E., Romeo M. (2022). The potential role of gut microbiota in Alzheimer’s disease: from diagnosis to treatment. *Nutrients*.

[21] Goyal D., Ali S. A., Singh R. K. (2021). Emerging role of gut microbiota in modulation of neuroinflammation and neurodegeneration with emphasis on Alzheimer's disease. *Progress in Neuropsychopharmacology & Biological Psychiatry*.

[22] Liu S., Gao J., Zhu M. Q., Liu K. D., Zhang H. L. (2020). Gut microbiota and dysbiosis in Alzheimer's disease: implications for pathogenesis and treatment. *Molecular neurobiology*.

[23] Doulberis M., Kotronis G., Gialamprinou D. (2021). Alzheimer’s disease and gastrointestinal microbiota; impact of *Helicobacter pylori* infection involvement. *International Journal of Neuroscience*.

[24] Kesika P., Suganthy N., Sivamaruthi B. S., Chaiyasut C. (2021). Role of gut-brain axis, gut microbial composition, and probiotic intervention in Alzheimer's disease. *Life Sciences*.

[25] Hung C. C., Chang C. C., Huang C. W., Nouchi R., Cheng C. H. (2022). Gut microbiota in patients with Alzheimer’s disease spectrum: a systematic review and meta-analysis. *Aging (Albany NY)*.

[26] Haran J. P., Bhattarai S. K., Foley S. E. (2019). Alzheimer's disease microbiome is associated with dysregulation of the anti-inflammatory P-glycoprotein pathway. *mBio*.

[27] Zhang M., Zhao D., Zhou G. H., Li C. B. (2020). Dietary pattern, gut microbiota, and Alzheimer's disease. *Journal of agricultural and food chemistry*.

[28] Wang X.-R., Shi G.-X., Yang J.-W. (2015). Acupuncture ameliorates cognitive impairment and hippocampus neuronal loss in experimental vascular dementia through Nrf 2-mediated antioxidant response. *Free Radical Biology & Medicine*.

[29] Forbes D., Forbes S. C., Blake C. M., Thiessen E. J., Forbes S. (2015). Exercise programs for people with dementia. *The Cochrane database of systematic reviews*.

RETRACTED

[30] Lee M. S., Shin B.-C., Ernst E. (2009). Acupuncture for Alzheimer's disease: a systematic review. *International Journal of Clinical Practice*.

[31] Kelly R. B., Willis J. (2019). Acupuncture for pain. *American Family Physician*.

[32] Lu L., Zhang X. G., Zhong L. L. D. (2016). Acupuncture for neurogenesis in experimental ischemic stroke: a systematic review and meta-analysis. *Scientific reports*.

[33] Chen Y. M., Xie X. L., Xiao P. Y. (2020). Acupuncture on treating asthma. *Medicine (Baltimore)*.

[34] Song G. Q., Fiocchi C., Achkar J. P. (2019). Acupuncture in inflammatory bowel disease. *Inflammatory Bowel Diseases*.

[35] Tan W., Lin S. C. (2020). Research progress on the mechanism of acupuncture and moxibustion in treating Alzheimer's disease. *Mod Tradit Chin Me Mater Med-World Sci Technol*.

[36] Lu W. D., Clower E. D., Gilman A. D., Rosenthal D. S. (2008). The value of acupuncture in cancer care. *Hematology/Oncology Clinics of North America*.

[37] Dean-Clower E., Doherty-Gilman A. M., Keshaviah A. (2010). Acupuncture as palliative therapy for physical symptoms and quality of life for advanced cancer patients. *Integrative Cancer Therapies*.

[38] Vinjamury S. P., Li J. T., Hsiao E. (2013). Effects of acupuncture for cancer pain and quality of life - a case series. *Chinese Medicine*.

[39] Li X., Guo F., Zhang Q. (2014). Electroacupuncture decreases cognitive impairment and promotes neurogenesis in the APP/PS1 transgenic mice. *BMC Complementary and Alternative Medicine*.

[40] Cao J., Tang Y. S., Li Y. J., Gao K., Shi X. D., Li Z. G. (2017). Behavioral changes and hippocampus glucose metabolism in APP/PS1 transgenic mice via electro-acupuncture at governor vessel acupoints. *Frontiers in Aging Neuroscience*.

[41] Wang X., Miao Y., Abulizi J. (2016). Improvement of electroacupuncture on APP/PS1 transgenic mice in spatial learning and ,memory probably due to expression of A<i>*β*</i> and LRP1 in hippocampus. *Evidence-based complementary and alternative medicine: eCAM*.

[42] Grienberger C., Rochefort N. L., Adelsberger H. (2012). Staged decline of neuronal function in vivo in an animal model of Alzheimer's disease. *Nature Communications*.

[43] Keskin A. D., Kekuš M., Adelsberger H. (2017). BACE inhibition dependent repair of Alzheimer's pathophysiology. *Proceedings of the National Academy of Sciences of the United States of America*.

[44] Radde R., Bolmont T., Kaeser S. A. (2006). Abeta 42-driven cerebral amyloidosis in transgenic mice reveals early and robust pathology. *EMBO reports*.

[45] Ferguson S. A., Sarkar S., Schmued L. C. (2013). Longitudinal behavioral changes in the APP/PS1 transgenic Alzheimer's disease model. *Behavioural Brain Research*.

RETRACTED

[46] Liu W., Zhuo P., Li L. (2017). Activation of brain glucose metabolism ameliorating cognitive impairment in APP/PS1 transgenic mice by electroacupuncture. *Free Radical Biology and Medicine*.

[47] Ma J., Gao Y., Jiang L. (2017). Fluoxetine attenuates the impairment of spatial learning ability and prevents neuron loss in middle-aged APPswe/PSEN1dE9 double transgenic Alzheimer's disease mice. *Oncotarget*.

[48] Langille M. G., Zaneveld J., Caporaso J. G. (2013). Predictive functional profiling of microbial communities using 16S rRNA marker gene sequences. *Nature biotechnology*.

[49] Kanehisa M., Goto S., Sato Y., Furumichi M., Tanabe M. (2012). KEGG for integration and interpretation of large-scale molecular data sets. *Nucleic acids research*.

[50] Parks D. H., Tyson G. W., Hugenholtz P., Beiko R. G. (2014). STAMP: statistical analysis of taxonomic and functional profiles. *Bioinformatics*.

[51] Nelson P. T., Jicha G. A., Schmitt F. A. (2007). Clinicopathologic correlations in a large Alzheimer disease center autopsy cohort: neuritic plaques and neurofibrillary tangles" do count" when staging disease severity. *Journal of Neuropathology and Experimental Neurology*.

[52] Kinney J. W., Bemiller S. M., Murtishaw A. S., Leisgang A. M., Salazar A. M., Lamb B. T. (2018). Inflammation as a central mechanism in Alzheimer's disease. *Alzheimers & Dementia*.

[53] La Joie R., Visani A. V., Baker S. L. (2020). Prospective longitudinal atrophy in Alzheimer's disease correlates with the intensity and topography of baseline tau-PET. *Science Translational Medicine*.

[54] Gouras G. K., Tsai J., Naslund J. (2000). Intraneuronal A*β*42 accumulation in human brain. *The American journal of pathology*.

[55] Martikainen I. K., Kemppainen N., Johansson J. (2019). Brain *β*-amyloid and atrophy in individuals at increased risk of cognitive decline. *AJNR American Journal of Neuroradiology*.

[56] GM M. K., Knopman D. S., Chertkow H. (2011). The diagnosis of dementia due to Alzheimer's disease: recommendations from the National Institute on Aging-Alzheimer's Association workgroups on diagnostic guideline s for Alzheimer's disease. *Alzheimer's & Dementia: The Journal of the Alzheimer's Association*.

[57] Szczepanik A. M., Funes S., Petko W., Ringheim G. E. (2001). IL-4, IL-10 and IL-13 modulate A beta (1-42)-induced cytokine and chemokine production in primary murine microglia and a human monocyte cell line. *Journal of neuroimmunology*.

[58] Michaud J. P., Rivest S. (2015). Anti-inflammatory signaling in microglia exacerbates Alzheimer's disease-related pathology. *Neuron*.

[59] Glass C. K., Saijo K., Winner B., Marchetto M. C., Gage F. H. (2010). Mechanisms underlying inflammation in neurodegeneration. *Cell*.

RETRACTED

[60] Guillot-Sestier M. V., Doty K. R., Gate D. (2015). IL10 deficiency rebalances innate immunity to mitigate Alzheimer-like pathology. *Neuron*.

[61] Li X. Z., Long J. T., He T. G., Belshaw R., Scott J. (2015). Integrated genomic approaches identify major pathways and upstream regulators in late onset Alzheimer's disease. *Scientific reports*.

[62] Zhang B., Gaiteri C., Bodea L. G. (2013). Integrated systems approach identifies genetic nodes and networks in late-onset Alzheimer's disease. *Cell*.

[63] Maldonado R. F., Sá-Correia I., Valvano M. A. (2016). Lipopolysaccharide modification in Gram-negative bacteria during chronic infection. *FEMS microbiology reviews*.

[64] Lukiw W. J. (2016). Bacteroides fragilis lipopolysaccharide and inflammatory signaling in Alzheimer's disease. *Frontiers in Microbiology*.

[65] Zhao Y., Zhao H., Lobo N., Guo X. Y., Gentleman S. M., Ma D. Q. (2014). Celastrol enhances cell viability and inhibits amyloid-*β* production induced by lipopolysaccharide in vitro. *Journal of Alzheimers Disease*.

[66] Wu D., Zhang X., Zhao M., Zhou A. L. (2015). The role of the TLR4/NF-*κ*B signaling pathway in A*β* accumulation in primary hippocampal neurons. *Sheng Li Xue Bao*.

[67] Kitazawa M., Oddo S., Yamasaki T. R., Green K. N., LaFerla F. (2005). Lipopolysaccharide-induced inflammation exacerbates tau pathology by a cyclin-dependent kinase 5-mediated pathway in a transgenic model of Alzheimer's disease. *The Journal of neuroscience: the official journal of the Society for Neuroscience*.

[68] Liu J., Wang D., Li S. Q., Yu Y., Ye R. D. (2016). Suppression of LPS-induced tau hyperphosphorylation by serum amyloid A. *Journal of Neuroinflammation*.

[69] Zhao Y. H., Jaber V., Lukiw W. J. (2017). Secretory products of the human GI tract microbiome and their potential impact on Alzheimer's disease (AD): detection of lipopolysaccharide (LPS) in AD hippocampus. *Frontiers in cellular and infection microbiology*.

[70] Lu J., Guo P., Liu X. (2019). Herbal formula Fo Shou San attenuates Alzheimer's disease-related pathologies via the gut-liver-brain axis in APP/PS1 mouse model of Alzheimer's disease. *Evidence-based complementary and alternative medicine: eCAM*.

[71] Song Q., Hu S., Wang H. B. (2014). Electroacupuncturing at Zusanli point (ST36) attenuates pro-inflammatory cytokine release and organ dysfunction by activating cholinergic anti-inflammatory pathway in rat with endotoxin challenge. *African journal of traditional, complementary, and alternative medicines: AJTCAM*.

[72] Harach T., Marungruang N., Duthilleul N. (2017). Reduction of Abeta amyloid pathology in APPPS1 transgenic mice in the absence of gut microbiota. *Scientific reports*.

RETRACTED

[73] Zhuang Z. Q., Shen L. L., Li W. W. (2018). Gut microbiota is altered in patients with Alzheimer's disease. *Journal of Alzheimer's Disease*.

[74] Zhu F. Q., Li C. R., Chu F. N., Tian X. P., Zhu J. (2020). Target dysbiosis of gut microbes as a future therapeutic manipulation in Alzheimer's disease. *Frontiers in aging neuroscience*.

[75] Bhatia A. M., Maisonneuve J. F., Persing D. H., Knobler S. L., O'Connor S., Lemon S. M., Najafi M. (2004). Propionobacterium acnes and chronic diseases. *The Infectious Etiology of Chronic Diseases: Defining the Relationship, Enhancing the Research, and Mitigating the Effects*.

[76] Zhuang Z. H., Yang R. T., Wang W. X., Qi L., Huang T. (2020). Associations between gut microbiota and Alzheimer's disease, major depressive disorder, and schizophrenia. *Journal of Neuroinflammation*.

[77] Shen L., Liu L., Ji H. F. (2017). Alzheimer's disease histological and behavioral manifestations in transgenic mice correlate with specific gut microbiome state. *Journal of Alzheimer's Disease*.

[78] Rosenberg E., DeLong E., Lory S., Stackebrandt E., Thompson F. (2014). Other major lineages of bacteria and the archaea. *The Prokaryotes*.

[79] Wang X. L., Zeng J., Feng J. (2014). Helicobacter pylori filtrate impairs spatial learning and memory in rats and increases Î²-amyloid by enhancing expression of presenilin-2. *Frontiers in Aging Neuroscience*.

[80] Wang X. L., Zeng J., Yang Y. (2014). Helicobacter pylori filtrate induces Alzheimer-like tau hyperphosphorylation by activating glycogen synthase kinase-3*β*. *Journal of Alzheimer's Disease*.

[81] Sun Z. Z., Li X. Y., Wang S., Shen L., Ji H. F. (2020). Bidirectional interactions between curcumin and gut microbiota in transgenic mice with Alzheimer's disease. *Applied microbiology and biotechnology*.

[82] Cattaneo A., Cattane N., Galluzzi S. (2017). Association of brain amyloidosis with pro-inflammatory gut bacterial taxa and peripheral inflammation markers in cognitively impaired elderly. *Neurobiology of Aging*.

[83] Hsiao E. Y., McBride S. W., Hsien S. (2013). Microbiota modulate behavioral and physiological abnormalities associated with neurodevelopmental disorders. *Cell*.

[84] Zhang L., Wang Y., Xiayu X. (2017). Altered gut microbiota in a mouse model of Alzheimer's disease. *Journal of Alzheimer's Disease*.

[85] Rezaeiasl Z., Salami M., Sepehri G. (2019). The effects of probiotic and strains on memory and learning behavior, long-term potentiation (LTP), and some biochemical parameters in *β*-amyloid-induced rat's model of Alzheimer's disease. *Preventive Nutrition and Food Science*.

RETRACTED

[86] Claesson M. J., Jeffery I. B., Conde S. (2012). Gut microbiota composition correlates with diet and health in the elderly. *Nature*.

[87] Liang S., Wang T., Hu X. (2015). Administration of Lactobacillus helveticus NS8 improves behavioral, cognitive, and biochemical aberrations caused by chronic restraint stress. *Neuroscience*.

[88] Wang T., Hu X., Liang S. (2015). Lactobacillus fermentum NS9 restores the antibiotic induced physiological and psychological abnormalities in rats. *Beneficial Microbes*.

[89] Wu L., Han Y. Q., Zheng Z. P. (2021). Altered gut microbial metabolites in amnestic mild cognitive impairment and Alzheimer’s disease: signals in host–microbe interplay. *Nutrients*.

[90] Udhayabanu T., Manole A., Rajeshwari M., Varalakshmi P., Houlden H., Ashokkumar B. (2017). Riboflavin responsive mitochondrial dysfunction in neurodegenerative diseases. *Journal of Clinical Medicine*.

[91] Xie K., Qin Q., Long Z. P. (2021). High-throughput metabolomics for discovering potential biomarkers and identifying metabolic mechanisms in aging and Alzheimer’s disease. *Frontiers in Cell and Developmental Biology*.

[92] Madeira C., Vargas-Lopes C., Brandão C. O. (2018). Elevated glutamate and glutamine levels in the cerebrospinal fluid of patients with probable alzheimer's disease and depression. *Frontiers in Psychiatry*.

[93] He Y., Wang Y. M., Liu S. (2020). A metabolomic study of the urine of rats with Alzheimer's disease and the efficacy of Ding-Zhi-Xiao-Wan on the afflicted rats. *Journal of Separation Science*.

[94] Liang Q., Liu H., Lia X., Zhang A. H. (2016). High-throughput metabolomics analysis discovers salivary biomarkers for predicting mild cognitive impairment and Alzheimer's disease. *Rsc Advances*.

